# Persistence of COVID-19 Human Milk Antibodies After Maternal COVID-19 Vaccination: Systematic Review and Meta-Regression Analysis

**DOI:** 10.7759/cureus.59500

**Published:** 2024-05-02

**Authors:** Naema I Hamouda, Ahmed Mostafa Amin, Mohammed T Hasan, Ehssan Baghagho

**Affiliations:** 1 Neonatology, El-Sahel Teaching Hospital/General Organization for Teaching Hospitals and Institutes, Cairo, EGY; 2 Internal Medicine, Faculty of Medicine, Al-Azhar University, Cairo, EGY; 3 Public Health, General Organization for Teaching Hospitals and Institutes, Cairo, EGY

**Keywords:** covid-19 vaccine, sars-cov-2 vaccine, antibody level, breast milk, human milk

## Abstract

The World Health Organization (WHO) declared COVID-19 a pandemic. The Centers for Disease Control and Prevention (CDC), WHO, and American College of Obstetricians and Gynecologists (ACOG) recommend vaccination of pregnant and lactating women, aiming to protect both mothers and their infants through transplacental and human milk antibody transmission. This study aims to assess the quantity of antibodies in human milk and determine the effect of time, vaccine type, and dose on antibody level. Single-arm prospective observational studies reporting the COVID-19-specific antibody level in human milk after COVID-19 vaccination during pregnancy or lactation were included. PubMed, Scopus, Cochrane, EBSCO, and Web of Science were searched from December 2019 to November 22, 2022. Data were extracted in a uniform Google sheet. A total of 2657 studies were identified. After the removal of duplicates and screening, 24 studies were included in the systematic review and meta-regression. Human milk COVID-19-specific antibody levels increased with subsequent vaccine doses, as reflected by a positive relationship for the second (coefficient=0.91, P-value 0.043 for IgA and coefficient=1.77, P-value 0.009 for IgG) and third (coefficient=1.23, P-value 0.0029 for IgA and coefficient=3.73, P-value 0.0068 for IgG) doses. The antibody level exhibited a weak positive relationship with the follow-up time (coefficient=0.13, P-value 0.0029 for IgA and coefficient=0.18, P-value 0.016 for IgG). Only one of the 38 infants showed detectable COVID-19 IgM and IgA antibody levels in their blood. There was an increase in the neutralizing activity of COVID-19 antibodies in human milk following the COVID-19 vaccination. From the analysis of published data, we found high positive levels of antibodies in human milk that increased with subsequent doses. Additionally, the human milk antibodies exhibit a positive neutralizing effect. Only one infant had detectable COVID-19 IgM+IgA antibodies in the blood. Further research is needed to discuss infant protection through a mother's vaccination.

## Introduction and background

In December 2019, the authorities in Wuhan, China, officially informed the World Health Organization (WHO) of the existence of numerous cases of a newly identified respiratory disease. China promptly confirmed the existence of a new pathogenic virus belonging to the *Coronaviridae* family. The complete genome of this coronavirus was made publicly available on January 28, 2020, and it was officially designated as COVID-19 by WHO on February 11 [1]. The severe acute respiratory syndrome coronavirus 2 (SARS-CoV-2) has rapidly spread worldwide, causing a disastrous disease in humans known as coronavirus disease 2019 or COVID-19. This disease has had an enormous impact not only on global health but also on the economy [2].

The COVID-19 pandemic shifted research priorities, and since then, developing reliable and effective vaccines has become a global hope. Administering preventive strategies against infection and finding cures to lessen the symptoms have become a primary research concern [3,4].

Diverse vaccines for COVID-19 have been licensed. These include the mRNA-based COVID-19 vaccine (Pfizer-BioNTech and Moderna) [5], the adenovirus-based vector vaccine (Johnson & Johnson and Oxford-AstraZeneca) [6], and the recombinant viral vector vaccine (CanSino Biologics) [7].

As per the established guidelines for clinical trials, COVID-19 vaccines initially did not include trials in pregnant and/or lactating women. However, later on, the Centers for Disease Control and Prevention (CDC), WHO, and the American College of Obstetricians and Gynecologists (ACOG) recommended the vaccination of all eligible people, including pregnant women or those in the postpartum period [8,9]. Furthermore, it has been shown that vaccination can promote passive immunization in infants and provide a first line of defense against different pathogens.

Breast milk is the best source of nutrition and immunity through the transmission of antibodies, either following a natural infection or vaccination [10]. Breast milk is composed of a wealth of specific immune-protective factors. Among these, human milk antibodies comprise largely secretory immunoglobulins A (IgA, >90%), as well as secretory immunoglobulins M (IgM, 8%) and immunoglobulins G (IgG, 2%) [11].

Previous systematic reviews have discussed the safety, acceptance, and effectiveness of the COVID-19 vaccine and the existence of COVID-19 antibodies in human breast milk following SARS-CoV-2 vaccination among pregnant and lactating women. The focus primarily revolved around mRNA vaccines [12-15]. Only one meta-analysis was conducted on the presence of COVID-19 antibodies in human milk without discussing the effect of time, type of vaccine, and the number of vaccine doses on the antibody levels [16].

Therefore, the aim of this study was to assess the quantity of COVID-19-specific antibodies in human milk and determine the effect of time, vaccine type, and the number of doses on the COVID-19-specific antibody level.

## Review

Methods

We followed the Preferred Reporting Items for Systematic Review and Meta-Analysis 2020 (PRISMA) criteria in conducting this systematic review and meta-analysis [17]. We prospectively registered our study on the PROSPERO database (CRD42023439229).

Eligibility Criteria and Selection Process

Two independent authors (NH and EB) conducted a comprehensive search on the following databases: Scopus, PubMed, Cochrane, EBSCO, and Web of Science. We used the following search strategy: (SARS-CoV-2 vaccine) OR (COVID-19 vaccine) AND (breast milk) AND (antibody level). We then uploaded all the identified records on the Rayyan website, and duplicates were removed using Rayyan [18]. Then, we assessed the remaining studies for eligibility.

We included single-arm prospective observational studies that met the following criteria: (1) their population is breastfeeding women who were vaccinated or decided to be vaccinated against COVID-19 during pregnancy or breastfeeding by any available vaccine and with any number of doses; and (2) studies that measure COVID-19-specific antibody levels (IgA, IgG, or IgM) in milk and their persistence throughout time. The exclusion criteria were case reports, case series, double-arm studies, studies on antibodies against human coronaviruses (including SARS-CoV-2), and those searching for COVID-19 viral particles in human breast milk. We screened the studies in two steps. First, title and abstract screening by Rayyan and then full-text screening. We also screened the references of all the studies included in the full-text screening. The screening was done by two independent authors (AM and EB), and disagreement was resolved by the third author (NH).

Data Extraction and Quality Assessment

Two independent authors (AM and EB) extracted the data into a uniform Google sheet, and any disagreement was resolved by the third author (NH). The following data were extracted: (1) a summary of included studies, (2) population characteristics of included studies, and (3) primary and secondary outcomes.

The Newcastle-Ottawa scale was used to assess the risk of bias in the included studies by two independent authors (AM and EB), which included the following domains: (1) Selection, (2) Comparability, and (3) Outcome. The study was judged to be of good quality if it got three or four stars in the selection domain and one or two stars in the comparability domain and two or three stars in the outcome domain. The study was considered of fair quality if it deserved two stars in the selection domain and one or two stars in the comparability domain and two or three stars in the outcome domain. The study was reported to be of poor quality if it gets zero or one star in the selection domain or zero star in the comparability domain or zero or one star in the outcome domain [19].

Data Analysis

According to our data, the units of measurement were completely different, and there was no statistical way to convert them to each other. We used log-transformed mean to reduce variance and skewness in the data [20,21]. We used a meta-regression model to test the effect of the vaccine type, number of doses, and time on COVID-19-specific antibody levels in human milk using the R software (R Foundation for Statistical Computing, Vienna, Austria) version 1.4.1717, R-4.3.2 for Windows. Different units of measurement do not affect the meta-regression model [22]. We assessed the level of heterogeneity using I2 and chi-square test; significant heterogeneity was considered when chi-square P<0.1. Time was measured in weeks. For studies that report time in range, we took the mean of the time range.

Results

A total of 2633 studies were identified through PubMed, Cochrane, Web of Science, Scopus, and EBSCO, which were then uploaded to Rayyan. An additional 25 studies were added from manual screening. After the removal of duplicates by Rayyan, 2106 articles were screened for eligibility. We excluded 2006 studies based on the exclusion criteria during the title and abstract screening, and another 80 studies were excluded in the full-text screening step. We included only single-arm studies. Finally, we included 24 studies in our systematic review, and only 19 were eligible for the meta-analysis. The PRISMA flow diagram is shown in Figure 1 [23].

**Figure 1:** The Preferred Reporting Items for Systematic Review and Meta-Analysis (PRISMA) flow diagram.

Characteristics of the Included Studies

All the included studies were longitudinal prospective observational studies, comprising 824 women. In 21 studies, the mothers received the vaccine postpartum. Only three studies included women who received the vaccine during pregnancy. Eighteen studies reported the use of mRNA COVID-19 vaccines, specifically Pfizer or Moderna vaccines, and two of them reported the use of three doses of Pfizer. Four studies reported the use of four available COVID-19 vaccines (Pfizer, Moderna, Janssen, AZ). Previous SARS-CoV-2 infection was reported only in four studies in a range of 3%-13% of participants, while five studies did not report the state of prior infection. There was variability in the timeline of human milk COVID-19-specific antibody measurement that ranged from one month up to nine months from the first dose and only one study up to three months after the Pfizer vaccine booster dose. The summary of studies and patient characteristics is shown in Tables 1, 2.

**Table 1:** Summary of the included studies. *mean (range). Anti-RBD, anti-receptor-binding domain; NA, not available; IgG, immunoglobulin G; IgM, immunoglobulin M; IgA, immunoglobulin A; OD, optical density; AU/ml, arbitrary unit/ml; AZ, AstraZeneca; J&J, Johnson & Johnson; HCW, healthcare worker.

Study ID	Country, Study Design	Participant, Number	Maternal Age (y)	Postpartum Time (m)	Previous SARS-CoV-2 Infection, n (%)	Main Outcome	Unit of Measurement	Time Points
Bender et al. [24]	USA Cohort Single	Pregnant or lactating women vaccinated 3 doses Pfizer, 1 received J&J (n=10)	35.1 (30.9-42.8)*	NA	0	Anti-RBD IgG, IgM, IgA in breast milk. Maternal serum IgA, IgG. Correlation between maternal serum & breast milk antibody level. Neutralizing activity	OD490	Pre-vaccination, 1, 3, 6, 9 post-1st dose, and 1 month post-3rd dose
Baird et al. [25]	USA Cohort Single	HCW lactating women received Moderna or Pfizer (n=7)	NA	NA	NA	Anti-spike, anti-RBD IgA, IgG antibodies in human milk	U/ml	Pre-vaccination, 1, 4, 7, 11, 14 days post-1st and 2nd dose
Calil et al. [26]	Brazil Prospective Single	Lactating vaccinated with 2 doses of Sinovac (n=16)	35.6±3.2	11.2±8.7	0	Anti-SARS-CoV-2 IgA antibody in human milk	Ratio	Pre-vaccination and weekly after 1st dose until 7 weeks then at 4 months after 1st dose
Esteve-Palau et al. [27]	Spain Cohort Single	HCW lactating more than 18 years vaccinated with Pfizer-BioNTech 2 doses (n=33)	37.4±3.3	17.5±10.1	0	Anti-spike (S1) IgG antibody in human milk and its correlation to maternal serum level	AU/ml	2 weeks after 1st dose, 2,4, 12, and 24 weeks after 2nd dose
Henle [28]	USA Prospective Across USA	Pregnant/lactating women received 2 doses of Pfizer vaccine 6 months before study entry then receive 3rd dose (n=12)	35.45±4.17	3.58±1.8 (pregnant) 10.84±0.64 (lactating)	0	Anti-RBD IgG & IgA in breast milk following booster dose of Pfizer vaccine	U/ml	30 days and 1 day pre-booster, and 7, 14, 21, 30, 45, and 60 days
Juncker et al. [29]	Netherlands Cohort Single	Lactating women received mRNA-based COVID-19 vaccine BNT162b2, 20 received 2 doses and 6 only 1 dose (n=26)	33.28±3.14	7±3.137	1 (3.8%)	Anti-spike IgA antibody in human milk and IgG in maternal serum	OD450	Pre-vaccination, 3, 5, 7, 9, 11, 13, and 15-17 days after 1st and 2nd dose
Juncker et al. [30]	Netherlands Cohort Single	Lactating women vaccinated with Pfizer, Moderna, or AZ COVID-19 vaccine. J&J (n=134) 2 doses	34±6.25 33.5±9.2 33±6.16 32±7.86	7.5±7.03 5.2±6.13 5.2±7.7 4.5±6.6	1 2 2 2	SARS-CoV-2 IgA, IgG antibodies in human milk and IgG in maternal serum	OD450	Pre-vaccination, 3, 5, 7, 9, 11, 13, and15-17 days after 1st and 2nd dose. Last sample 56-84 days after G&G. 98 days after AZ
Kelly et al. [31]	USA Prospective Single	Lactating vaccinated 2 doses of Pfizer (n=5)	33±6.28	9.8±8.7	NA	Anti-spike IgG and IgA immunoglobulins in human milk	OD450	Pre-vaccination, 10-19, 20-29, 30-39, 40 days or more post-1st dose
Lebbe et al. [32]	Belguim Cohort Single	Lactating vaccinated women 2 doses(Pfizer) n=12	31.8±12.6	9.91±7.95	0	Anti-spike protein IgG, IgM, and IgA in maternal serum breast milk and infant serum	AU/ml	4 and 8 weeks after 1st dose
Narayanaswamy et al. [33]	USA Cohort Single	Lactating women received 2 doses of BNT-162b2 (Pfizer-BioNTech) or mRNA-1273 (Moderna) (n=30)	35.7 (26-46)*	10.1 (0.25-21.7)	Pfizer 2 (10%). Moderna 1 (10%)	Detection of anti-RBD IgA, IgG antibodies in human milk	OD450	Pre-vaccination and 3 weeks post-2nd dose
Perl et al. [34]	Israel Cohort Across Country	HCW women lactating receiving 2 doses Pfizer (n=84)	34±4	10.32±7.31	NA	Anti-SARS-CoV-2 IgA and IgG antibody in breast milk	U/ml	Pre-vaccination, 2, 3, 4, 5, and 6 weeks after 1st dose
Perez et al. [35]	USA Prospective Single	Pregnant & lactating women vaccinated 2 doses of Pfizer 26 or Moderna 3 (n=30)	34.9 (27.1-43.3)*	NA	4 (13.3%)	SARS-CoV-2 specific antibodies in serum and breast milk, neutralizing activity, effect of Pasteurization & persistence through 6 months after vaccination	OD490	Pre-vaccination, 1, 3, and 6 months after 1st dose
Rosenberg-Friedman et al. [36]	Israel Cohort Single	HCW lactating vaccinated received 2 doses of Pfizer (n=10)	34.6 (30-38)*	5.13±2.88	NA	Anti-spike and RBD-specific IgG and IgA in maternal serum and breast milk. Neutralization capacity of breast milk antibodies	End point titer	7 and 14 days after 1st and 2nd dose
Ricaadi et al. [37]	Italy Prospective Single	HCW lactating vaccinated 2 doses of Pfizer (n=18)	34±4.5	11.5±8.5	0	Pre-vaccination, pre-1st dose, 3 weeks after 2nd dose, and 6 months after 1st dose	AU/ml	Anti-SARS-CoV-2 spike (S) IgG & IgA in breast milk and maternal serum
Sajadi et al. [38]	USA Cross-Sectional Cohort Single	Pregnant women (n=10), breastfeeding mothers (n=12) Pfizer or Moderna 13.6% received 2 doses	32.6±3.2 34.2±3.4	NA 12±3.42	0	Anti-spike protein IgA and IgG in mother blood, breast milk, baby blood, nose, and stool	End point titer	36.7 weeks after 1st dose, 24.6 weeks after 1st dose
Trofin et al. [39]	Romania Prospective Single	Lactating vaccinated 2 doses of Pfizer 23/ Moderna 3 (n=26)	33.1±2.38	4.61±3.4	0	Measure the IgA and IgG anti-SARS-CoV-2 RBD titer in breast milk	U/ml	30 and 60 days after 2nd dose
Valcarce et al. [40]	USA Prospective Single	HCW lactating vaccinated 2 doses of Pfizer 14 or Moderna 7 (n=21)	34±3.9	6.8±4.8	0	Levels of anti-SARS-CoV-2 IgA and IgG in human milk and plasma	U/ml	Pre-vaccination, 15-30 days post-1st dose, 7-10 days post-2nd dose
Yeo et al. [41]	Singapore Cohort Single	HCW lactating women received 2 doses of BNT162b2 vaccine (n=35)	34±3.09	8.78±6.96	0	Neutralizing activity of antibodies in maternal serum & breast milk, SARS-CoV-2 spike RBD-specific antibody	OD450	Pre-vaccination, 1, 3, 7, 14, 21 after both vaccine doses
Yang et al. [42]	USA Cohort Multicenter	Lactating women were scheduled to be or had recently been vaccinated with 2 doses of Pfizer, Moderna, or AZ COVID-19 vaccine. J&J (n=54)	NA	NA	0	Anti-spike IgG, IgA in human milk	OD450	1 week before vaccination and 14 days for Pfizer/Moderna/AZ or 21–35 days (J&J) after completion of the vaccine regimen

**Table 2:** Summary of the studies that were not included in the meta-regression analysis. NA, not available; J&J, Johnson & Johnson; PEG, polyethylene glycol; IgG, immunoglobulin G; IgM, immunoglobulin M; IgA, immunoglobulin A.

Author, Year	Country, Study Design	Reason of Exclusion	Participant (n)	Maternal Age (y)	Postpartum Time (m)	Previous SARS-CoV-2 Infection, n (%)	Main Outcome	Time Points
Juncker et al. [43]	Netherlands Prospective Single	Results were reported as % of participant with detectable level of COVID-19-specific human milk antibody	Lactating women received full vaccination of one of four types of vaccines (n=124)	NA	NA	0	IgA antibody response in human milk (% of participants with detectable IgA, IgG)	Pre-vaccination, 20, 40, 60, 80, 100 days after 1st dose
Golan et al. [44]	USA Cohort Single	Graphical presentation of the results that cannot be extracted	Lactating women received Pfizer or Moderna vaccine (n=48)	35.6±3.8	5.8±4.5	NA	Anti-SARS-CoV-2 in human milk and maternal serum PEGylated proteins in human milk. Vaccine-related symptoms	Pre-vaccination, pre-2nd dose, 4-10 weeks after 2nd dose
Guida et al. [45]	Italy Cohort Single	Antibody measured as a whole not categorized as IgG, IgA, or IgM	Lactating women received 2 doses of Pfizer vaccine (n=10)	34.8±4.2	11±5.1	0	Anti-spike antibody (total) in human milk and maternal serum	Pre-vaccination and 7 days after 2nd dose
Stafford et al. [46]	USA Cohort Single	Results were reported as geometric mean	Lactating women received Moderna mRNA-1273. Pfizer-BioNTech BNT162b2. J&J (n=36)	33.5±3.9	5.2±6.2	1 (3%)	Level of anti-SARS-CoV-2-IgA, IgG-specific antibodies in breastfeeding infants’ stools, mother’s plasma, and human milk following maternal vaccination. Neutralizing capacity of antibody	Pre-vaccination, 15-30 days after 1st dose, 7-30 days, 60-75 days, 90-105 days, and 6 months after 2 doses of vaccine
Sadiq and Arslan [47]	Pakistan Cross-sectional Cohort Single	Results were reported as mean only	Lactating mother received 2 doses of Sinopharm or Sinovac (n=21)	31 (24-38)	17 (10-24)	0	Anti-spike IgG antibody in human milk and maternal serum	Pre-vaccination and 21 days after 2nd dose

According to the Newcastle-Ottawa quality assessment scale, in the selection domain, all studies were considered good or fair quality except for Calil et al., Kelly et al., Rosenberg-Friedman et al., and Perez et al. [26,31,35,36]. In the comparability domain, all studies were considered low quality due to the inclusion of single-arm studies. Therefore, it would be unfair to judge these studies according to the comparability domain. In the outcome domain, all studies are considered high quality except for Juncker et al. [29] due to a short follow-up time and inadequate follow-up data (Figure 2) [19].

**Figure 2:** Quality assessment using the Newcastle-Ottawa quality assessment scale

Human Milk COVID-19-Specific Antibody Level

We used meta-regression to test the effect of the COVID-19 vaccine on human milk antibody levels in relation to vaccine dose, time, and type of vaccine. The level of COVID-19-specific antibodies in human milk remained consistent over time and increased with subsequent doses (Table 3) (Figures 3, 4). There was a strong positive relationship between the Moderna vaccine and human milk COVID-19-specific antibody (coefficient=6.22, P-value <0.001 for IgA and coefficient=6.56, P-value <0.0001 for IgG). While for J&J, there was a weak positive relationship for IgA (coefficient=0.39, P-value 0.615) and a negative relationship for IgG (coefficient=-0.33, P-value 0.76) (Table 3).

**Table 3:** Meta-regression analysis. J&J, Johnson & Johnson; IgA, immunoglobulin A; IgG, immunoglobulin G.

		IgA	P-value	IgG	P-value
Vaccine dose	2nd dose	0.915	0.043	1.77	0.0092
	3rd dose	1.23	0.24	3.73	0.0068
Follow-up time		0.13	0.0029	0.18	0.016
Vaccine type	Moderna	6.22	<0.0001	6.56	<0.0001
	Pfizer	1.41	<0.0075	3.03	<0.0001
	Sinovac	1.02	0.21		
	J&J	0.39	0.615	-0.33	0.76

**Figure 3:** Human milk COVID-19-specific IgA antibody meta-regression analysis.

**Figure 4:** Human milk COVID-19-specific IgG antibody meta-regression analysis.

Five studies reported the use of any type of vaccine without reporting the results according to the type of vaccine. Therefore, we analyzed these studies separately. Human milk COVID-19-specific antibodies have a weak positive relationship with subsequent vaccine dose (coefficient=0.65, P-value 0.62 for IgA and coefficient=0.3, P-value 0.84 for IgG) and time (coefficient=0.035, P-value 0.28 for IgA and coefficient=0.079, P-value 0.023 for IgG) (Table 4). There was significant heterogeneity among studies regarding all outcomes, with an I2 value exceeding 99% (P-value>0.0001).

**Table 4:** Meta-regression analysis of the studies that report the antibody level without specification of the type of vaccine.

		IgA	P-value	IgG	P-value
Vaccine dose	2nd dose	0.65	0.62	0.3	0.84
Follow-up time		0.035	0.28	0.079	0.023

Level of Antibody in Infant Blood

Four studies investigated the presence of SARS-CoV-2-specific antibodies in 38 infant serums after mother immunization; only one of the 38 infants showed detectable anti-SARS-CoV-2 IgM+IgA antibodies [26,36,37,43].

Neutralizing Activity of Human Milk SARS-CoV-2 Antibody Following Vaccination

Five studies investigated the neutralizing activity of human milk antibodies post-SARS-CoV-2 vaccination. All these studies showed an increase in the neutralizing activity of human milk post-vaccination compared to pre-vaccination. With time, there was a decline in the neutralizing activity. Perez et al. showed a decrease of inhibition % activity with time to a level < cutoff value at six months post-vaccination. Stafford et al. showed low mean viral adherence to cells at six months (0.03) compared to pre-vaccination (0.14).

Discussion

We found an increase in the COVID-19-specific antibody levels in human milk with booster vaccine doses, which was reflected by a positive relationship for the second (coefficient=0.91, P-value 0.043 for IgA and coefficient=1.77, P-value 0.009 for IgG) and third (coefficient=1.23, P-value 0.25 for IgA and coefficent=3.73, P-value 0.0068 for IgG) vaccine doses. However, there is a weak positive relationship between time and both IgA and IgG. Notably, the Moderna vaccine has a strong positive relationship with human milk COVID-19-specific IgA and IgG antibody (coefficient=6.22 and 6.65), followed by the Pfizer vaccine (coefficient=1.41 and 3.03). In contrast, J&J has a weak positive relationship for IgA (coefficient=0.39) and negative relationship for IgG (coefficient=-0.33).

In terms of the antibody levels found in the infant's blood, the included studies indicate that the transfer of antibodies from the mother to the infant may not be sufficient to provide protection against SARS-CoV-2 infection. However, there was an increase in neutralizing activity of human milk COVID-19-specific antibodies post-vaccination compared to pre-vaccination, with a negative correlation between neutralizing activity and time.

Explanation of the Finding

The COVID-19 pandemic was a global crisis that affected every country worldwide. Pregnant and lactating women have an increased risk for COVID-19 infection and mortality [48]. Research has demonstrated that COVID-19 can be transmitted via the placenta and breast milk, potentially leading to complications associated with prematurity [49,50]. Therefore, it is crucial to protect infants through passive immunization. After the COVID-19 vaccine became available, further studies were conducted to show the beneficial effect of vaccination of pregnant and lactating women on infants. Studies showed that antibodies can be transmitted during pregnancy and breastfeeding, which explains the increase in antibody levels in breast milk post-vaccination. Therefore, it was recommended that all pregnant and lactating women be vaccinated [14,51]. Booster doses of vaccines can increase the reactogenicity in the recipient, which provides additional protection [51].

Agreement and Disagreement With Previous Studies

We have identified six previous systematic reviews and one systematic review with meta-analysis [13-15,49,52,53]. All of these studies agreed with our finding that there is an increase in the breast milk COVID-19-specific antibodies after vaccination, which could provide proper protection for the infant in the first six months of life. Moreover, COVID-19-specific IgG increases significantly after the second dose of the vaccine, which is consistent with our study [13,52,53]. Whited et al. analyzed the positivity rate of human milk COVID-19-specific antibodies. They concluded that there was an increase in antibody levels after vaccination, which is consistent with the result of our analysis [16]. None of the previous systematic reviews have assessed the correlation between antibody levels and time, nor have they compared the different vaccines included in our analysis.

Limitation

Our study has several limitations. Pregnant and lactating women were excluded from initial trials conducted to assess the efficacy and safety of the vaccines. Consequently, all the included studies were prospective observational studies that provided low-quality evidence. Due to the challenges provided by the pandemic, we have included only single-arm studies since it was difficult to find a control group that had not been exposed to COVID-19 or had been exposed but not vaccinated. The included studies exhibited a high tendency for bias due to their single-arm design. There were many differences in units of measure among the included studies, which increased the heterogeneity of the data. The generalizability of the results is difficult due to the small sample size of each included study.

## Conclusions

Our literature search indicates that vaccinating pregnant and lactating women can have positive effects on both the mother and infant, as it increases the antibody levels in breast milk, providing passive immunization to the infant. The dual or triple doses of vaccine further increase the COVID-19-specific human milk antibody levels compared to a single dose.

Well-conducted randomized controlled trials are essential to examine the duration of the persistence of antibodies in human milk and the long-term effect of the vaccine. Further research is needed to understand the factors influencing the transmission of antibodies and the immune response in infants after maternal COVID-19 immunization.
